# Large-Area Semiconducting Graphene Nanomesh Tailored by Interferometric Lithography

**DOI:** 10.1038/srep11463

**Published:** 2015-07-01

**Authors:** Alireza Kazemi, Xiang He, Seyedhamidreza Alaie, Javad Ghasemi, Noel Mayur Dawson, Francesca Cavallo, Terefe G. Habteyes, Steven R. J. Brueck, Sanjay Krishna

**Affiliations:** 1 Center for High Technology Materials, University of New Mexico, NM 87106, USA; 2 Department of Mechanical Engineering, University of New Mexico, NM 87131, USA; 3 Nanoscience and Microsystems Engineering, University of New Mexico, NM 87131, USA

## Abstract

Graphene nanostructures are attracting a great deal of interest because of newly emerging properties originating from quantum confinement effects. We report on using interferometric lithography to fabricate uniform, chip-scale, semiconducting graphene nanomesh (GNM) with sub-10 nm neck widths (smallest edge-to-edge distance between two nanoholes). This approach is based on fast, low-cost, and high-yield lithographic technologies and demonstrates the feasibility of cost-effective development of large-scale semiconducting graphene sheets and devices. The GNM is estimated to have a room temperature energy bandgap of ~30 meV. Raman studies showed that the G band of the GNM experiences a blue shift and broadening compared to pristine graphene, a change which was attributed to quantum confinement and localization effects. A single-layer GNM field effect transistor exhibited promising drive current of ~3.9 μA/μm and ON/OFF current ratios of ~35 at room temperature. The ON/OFF current ratio of the GNM-device displayed distinct temperature dependence with about 24-fold enhancement at 77 K.

Graphene has risen as a fascinating two-dimensional (2D) material for its high carrier mobility^1^, flexibility^2^, transparency^3^, and its extraordinary ability to withstand mechanical stress^4^. Due to these properties, graphene lends itself to many applications in electronics^5^,^6^, optoelectronics^7^,^8^, sensing, and energy storage^9^,^10^. However, graphene lacks a bandgap, which limits its application in digital electronics and optoelectronics. Extensive efforts^11^,^12^,^13^,^14^,^15^,^16^,^17^,^18^,^19^,^20^,^21^ have been made to create semiconducting graphene without disrupting its exceptional transport properties. One scheme is to obtain bandgap through quantum confinement in graphene nanoribbons (GNRs)^22^,^23^ and graphene nanomesh (GNM)^20^,^21^,^24^ with a critical dimension lower than 10 nm. These nanostructures enable potential applications of graphene in electronic and photonic devices, such as highly sensitive sensors^25^,^26^, in next-generation spintronics^27^,^28^, and in energy harvesting^29^,^30^ devices. Duan and co-workers^20^, fabricated semiconducting graphene using copolymer lithography and demonstrated that GNM-based field-effect transistors (FETs) exhibit comparable ON/OFF current ratios but 100 times higher drive currents than those of the similar devices based on individual GNRs. Furthermore, because of its excellent stability, 2D nature, and high electrical sensitivity, GNM is a good candidate to replace traditional solid-state nanoporours materials in fabrication of composite materials^31^ and electrochemical capacitors^32^ as well as in DNA sequencing^33^.

The fabrication of graphene nanomesh for practical applications demands efficient nanopatterning technologies to inexpensively produce nanoscale periodic modulations over large-areas. To our knowledge, a reliable technology with a wafer-scale fabrication capability for graphene nanomesh is still a challenge. E-beam lithography is a highly versatile technique to fabricate graphene nanostructures. However, it is not an economically viable approach when large-scale production is required^34^,^35^. Chemical methods, such as copolymer lithography^20^ and imprint lithography^36^ can meet the minimum feature size requirement, but they rely on rather complex operations, and are still limited to microscale areas^37^.

We demonstrate the use of interferometric lithography (IL)^38^,^39^,^40^,^41^,^42^,^43^,^44^ combined with oxygen (O_2_) plasma treatment to fabricate GNMs with sub-10 nm neck widths and high uniformity over a 1 × 1 cm^2^ area. Our approach is facile, inexpensive, and high throughput; furthermore it is based on well-established processing steps, which have been extensively characterized for decades. Finally our approach is compatible with the integrated circuits (IC) manufacturing technology^45^. In our work atomic force microscopy (AFM) and Raman spectroscopy were used to characterize the neck width of GNMs. The relative intensity of the D band increased with decreasing neck width. We also observed a blue shift and drastic broadening in the G band of the narrowest GNM, which can be attributed to the reduced size and edge effects. FETs with GNM channel widths of 2 mm were fabricated to demonstrate its application in electronic devices. Transfer characteristics of the GNM-device were studied at room and cryogenic temperatures. The GNM-FET with neck width of ~10 nm showed promising drive current values and ON/OFF current ratio at room temperature. Bandgap modulation was observed by tuning the source-drain voltage. In addition, the ON/OFF current ratio of the GNM-FET displayed distinct temperature dependence with a significant enhancement at 77 K.

## Results

Figure 1 illustrates the process flow for fabrication of the graphene nanomesh (GNM). We used commercially available single-layer (SL), chemical vapor deposited (CVD) graphene on a 285 nm silicon dioxide SiO_2_/p+ silicon substrate (Fig. 1a). The sample is spin-coated with negative photoresist (PR) and a square 2D hole array pattern is defined in the photoresist by IL (Fig. 1b and Methods). Subsequently, an isotropic O_2_ plasma etching is employed to reduce the PR neck width. In addition, the O_2_ plasma removes the unprotected graphene regions, which leads to a decrease in the graphene width still coated with PR (Fig. 1c). After the etching process, the PR is removed by soaking the sample in acetone to obtain the patterned GNM (Fig. 1d).

The narrow neck regions of the GNM strongly affect the charge transport through the structure^20^. Hence, the ability to precisely control the neck width is crucial for modulating the electronic properties in GNM. For GNMs made by IL, the neck width is tailored independently by varying the laser exposure dose and etching duration (Supplementary Information). We demonstrated the scalability of our approach by first making a highly uniform PR hole array pattern (serving as an etch mask) on three individual SL-CVD graphene samples and then performing O_2_ plasma etching on the processed samples for different time durations. The initial width and periodicity of the pattern transferred to the PR are ~70 nm and ~150–200 nm, respectively. Figure 2a,b show the cross section and top-view of a representative hole array mask. An optimized isotropic O_2_ plasma etching was carried out separately for 30, 60, and 80 seconds on the processed samples (see Methods). The corresponding SEM images are shown in Fig. 2(c–e). The cross-sectional SEM image in Fig. 2a reveals the corrugated sidewalls of the holes in the PR. Rough PR sidewalls are attributed to standing waves, resulting from the lack of an anti-reflection coating (ARC) layer. Therefore, a narrower GNM is expected compared to the hole array width on the PR surface. Figure 2g plots the average PR/GNM width as a function of etching time. A low magnification SEM image of the PR pattern on graphene after 80 seconds of etching is shown in Fig. 2f to show the uniformity of IL exposure and O_2_ plasma etch.

AFM images to characterize GNM neck-width were acquired from different regions of the GNM. GNMs with variable neck widths in the range of 6–20 nm are shown in Fig. 3a-c. More than 75% of the GNMs have neck widths between 8 nm and 12 nm. The standard deviation of the neck width is less than 3 nm over the entire GNM and the smallest measured neck width is ~7 ± 1 nm. The AFM height profile of a typical GNM (Supplementary Information) suggests that after the standard cleaning of the sample (see Methods), a thin PR residue ~15–20 nm is left on the graphene sheet, which potentially introduces some doping^46^ in the GNM and also affects the charge carrier mobility^47^ in the mesh structure. The nanomesh feature, with very minor breaks, was observed over the 1 × 1 cm^2^ wafer. The AFM profile studies on a set of samples with different etching durations (Supplementary Information) clearly revealed that highly uniform GNMs can be obtained with controllable neck widths using interferometric lithography.

## Discussion

In order to study the physical and electronic characteristics of the processed samples, GNMs with varying neck widths were characterized using Raman spectroscopy (see Methods). The Raman spectrum acquired from unpatterned graphene (Fig. 4a, black line) shows the G band centered at 1587 cm^−1^, which corresponds to the stretching vibration of carbon atoms^48^. Also a symmetric 2D band of the double resonance process^48^ is found centered at 2685 cm^−1^ with a full width at half-maximum (FWHM) of 32 cm^−1^. For the unpatterned graphene, only a low-intensity or no D band was observed. In contrast, for GNMs with varying neck widths, we observe an increase in the relative intensity of the D band (centered at 1352 cm^−1^) as the mesh neck width decreases (Fig. 4a). We attribute this feature to the increasing edge-to-surface ratio areas in samples with smaller neck widths^49^. The *I*_*D*_/*I*_*G*_ ratio of the unpatterned graphene and GNMs with different neck widths are shown in Fig. 4b. As shown in Fig. 4b, the G band characteristic of the GNM with 10 nm neck width is noticeably broader (10 cm^−1^) and blue shifted by 11 cm^−1^ compared to the G band dominating the spectrum of unpatterned graphene. This trend may be attributed to quantum confinement or localization effects resulting from edge disorders such as variable edge roughness in GNM^50^,^51^,^52^. In addition the GNM mesh was patterned using O_2_ plasma under a condition that is known to form oxygen-containing functional groups in graphite^53^. Because oxygen is more electronegative than carbon, such functional groups are expected to withdraw π electrons of GNM (i.e., dope with holes) and that potentially can induce a blue shift in the G band^54^. However, for the GNM with neck widths of ~50 nm, no shift or broadening was observed (Fig. 4b), which suggests that the doping effect is less dominant. Also, because the narrowest GNM in this study has a sub-10 nm neck width, a non-negligible confinement effect is expected. To validate the observed behavior of the G-band, multiple Raman scans were performed at different locations across the narrowest GNM sample. Figure 4c (inset) shows plots of the G-band peaks acquired at four different locations on the sample. The results plotted in Fig. 4c show that all of the G band peaks tend to stay at approximately 1605 cm^−1^ by a maximum shift of 17 cm^−1^ with respect to the unpatterned graphene. Also, the measured FWHM of the G bands at the four locations are within a range of 42–47 cm^−1^, indicating that, on average, the G band of the GNM is 10 cm^−1^ broader than that of the unpatterned graphene. The blue shift and broadening of the G band for the narrowest GNM is likely due to the lateral quantum confinement and localization effects and/or chemical doping by functional groups on the GNM edges.

In order to study the transport characteristics of the GNM, a field-effect transistor (Supplementary Information) with the mesh structure serving as the conduction channel was fabricated (see Methods). Due to its 2D nature, the drive current of graphene devices, can be scaled up by increasing the device area. This is of great significance for realizing high-frequency devices with sufficiently high drive current in large circuits^55^. Since our IL technique enables the fabrication of GNMs over of 1 × 1 *cm*^2^ area, the channel length and width of the transistor are chosen to be 14 *μm* and 2 mm, respectively. Figure 5a shows a schematic representation of the GNM-FET. Plots of source-drain current (*I*_*d*_) as a function of gate voltage (*V*_*g*_) at a constant source-drain voltage (*V*_*ds*_) are shown in Fig. 5b. The SL GNM-device delivered ~3.9 μA/μm current with an ON/OFF current ratio of ~9 at *V*_*ds*_ = −1 V. This is due mainly to a large GNM conduction channel filled with high density graphene ribbons capable of driving high currents. Importantly, at *V*_*ds*_ = −100 mV, although the ON-state current density is reduced to ~2.5 μA/μm, the ON/OFF current ratio has increased up to ~35. The modulation of the ON/OFF current ratio by varying the source-drain voltage is a characteristic of the GNM as it has not been reported for pristine graphene devices^56^. The measured dependence of the ON/OFF current ratio on V_ds_ indicates the semiconducting nature of the GNM^22^. This behavior is attributed to the formation of an electronic bandgap in graphene as a result of quantum confinement, edge and localization effects^36^,^57^. The latter also suggests that the blue shift and broadening in the G band for the narrowest mesh is likely due to confinement and localization effects. Multiple minor conduction plateaus are found in the *I*_*d*_−*V*_*g*_ transfer curves (Fig. 5b), possibly due to the formation of electronic subbands in the GNM^36^. The *I*_*d*_−*V*_*ds*_ for the GNM transistor (Fig. 5c) is non-linear, regardless of the applied gate voltage. In addition, although the Fermi-level modulation by the gate voltage is present, no saturation regions of the *I*_*d*_−*V*_*ds*_ curves are observed. The ON-state current of the GNM-FET is approximately 9 orders of magnitude lower than the one measured for an unpatterned graphene device (Fig. 5d). The ON current obtained from the GNM-FET is comparable to the results obtained for few-layer GNM-FETs^36^,^37^,^58^, and it is considerably higher than the reported GNR-FETs with similar width^59^,^60^. Moreover, the gate voltage sweeping range in the GNM-device is found to be smaller than that of the unpatterned graphene device. This is attributed to an increased leakage through the gate oxide after patterning. The reduced level of current compared to the bulk device is determined by the limited current pathway and the introduction of edge defects. The comparison (Fig. 5d) also shows that the charge neutrality point for the GNM is shifted toward higher positive gate voltage regions. This phenomenon is attributed to the absorption of charged impurities at the graphene edges induced by oxidation during the O_2_ plasma treatment and polymer residues^61^. Despite the fact that absorption of charged impurities by graphene edge terminations in the GNM in principle plays a role in doping of the structure, its impact on the semiconductor behavior of the GNM (i.e. bandgap, ON/OFF ratio, etc.) could be affected by many different factors^62^. Such factors may include the type of doping, the position of the dopant with respect to the ribbon edges, the ribbon width, and type of ribbon symmetry (i.e. zigzag and armchair edges). Isolating these various effects would require further systematic investigations. The electronic properties of GNM made by IL along with neck-width and sheet coverage area are compared with previously reported results obtained using different processes in Table 1.

The overall current of the GNM displayed a significant temperature dependence (Fig. 6a), where back-gate modulation at *V*_*ds*_ = −1 *V* increased from ~9 at room temperature to ~215 at 77 K. The ON/OFF current ratio of FET-devices exponentially scales with the bandgap as *I*_*ON*_/*I*_*OFF*_ ∝ exp(−*E*_*g*_/*k*_*B*_*T*), where *k*_*B*_ is Boltzmann constant and *T* is the absolute temperature^63^. We speculate that, at very low temperatures, the carriers energy (*k*_*B*_*T* << *E*_*g*_) was not sufficient to tunnel through the gap or hop through edge states and therefore the OFF-current state drops markedly. This temperature dependence is in strong contrast to that observed in unpatterned graphene FETs, where the pristine graphene is semi-metallic with a zero bandgap, and the temperature dependence of the transfer curves was negligible (Supplementary Information). Moreover, we noticed that the current plateau features are more pronounced at lower temperatures. The plateau structures are highly reproducible under different thermal cycles, and they are more pronounced at temperatures below 120 K. The former change in the plateau peaks is attributed to either stronger charge hopping through a series of quantum dots or to conduction associated with multiple one dimensional (1D) subbands generated in the mesh structure at lower temperatures^59^.

The effective mobility of holes in the SL-GNM produced by IL are estimated to be ~80 cm^2^ V^−1^ s^−1^ and ~165 cm^2^ V^−1^ s^−1^ at room temperature and 77 K, respectively (see Methods and Supplementary Information). The charge carrier mobility in GNM is limited by intrinsic scattering, phonon scattering from the supporting substrate, impurity scattering, and line edge roughness (LER) scattering^60^,^64^. The contributions of these scattering mechanisms comparatively vary with the temperature, Fermi-level location, and the neck width of the graphene mesh^65^. Therefore, the observed increase in the hole carrier mobility of the GNM, suggests that the net scattering mechanism is less effective at lower temperatures. These calculated values are relatively higher than reported carrier mobilities for single and few layer GNMs with the same average neck width (Table 1)^21^,^58^. The electronic bandgap of GNMs inversely scales with the average neck width (*w*) by the experimentally derived equation *E*_*g*_ ~ *α*/*w*, where *α* is between 0.3 and 1.5 with unit [nm eV]^66^. Also the ON/OFF current ratio of GNM-FETs varies exponentially with the bandgap, as specified by the following equation 1:



Using the measured ON/OFF current ratio at various temperature and inverting Eq. 1 to calculate the bandgap, we estimate *E*_*g*_ = 30 meV for a GNM with an average neck width of ~10 nm. As shown in Table 1, this value is in the range of those previously reported in the literature for a GNM with a comparable ribbons width^21^,^58^.

In summary, we have proposed and demonstrated a simple yet effective approach to produce highly uniform graphene nanomesh structures with sub-10 nm neck width across 1 × 1 *cm*^2^ areas. The fabrication of GNM using IL is scalable and can be performed using standard top-down fabrication methods. The fabricated GNM exhibited a semiconducting behavior with an estimated bandgap ~30 meV. GNMs with various neck widths in the range of 50-10 nm have been fabricated on a macroscopic scale with an unprecedented level of control. Raman studies have shown a significant broadening and blue shift of the G band for the narrowest GNM. Such blue shift is attributed to quantum confinement effects. The GNM devices have been fabricated and they have shown drive currents ~3.9 μA/μm, ON/OFF current ratios ~35 at room temperature and ~215 at 77 K, and mobilities suitable for field- effective devices operating at room temperature. The availability of direct bandgap GNMs over large areas provides exciting opportunities for graphene-based photodetectors^67^ and highly interconnected graphene networks^68^. Further narrowing of the GNM neck width is indeed possible and requires optimization on the etching parameters (i.e. gas pressure, RF power, etc.) to provide a finer control over transition from 10 nm neck width to 5 nm. Additionally, state of the art techniques such as scanning transmission electron microscopy (STEM) or AFM with carbon nanotube (CNT) tip will offer a more precise characterization for narrower mesh structures. IL parameters could also be used as additional variables in the GNM fabrication. Specifically, the laser wavelength and incident angle could be adjusted to make a structure with smaller periodicities, which in turn improves the drive current of the GNM-device.

## Methods

### Device fabrication

High-quality SL CVD graphene wafers on 285 nm SiO_2_/+p Si substrate with 95% uniformity were prepared from Graphene Supermarket Inc. The GNM-FETs were fabricated using standard photolithography (Figure S2). The heavily p-doped Si substrate and thermally grown 285 nm-thick SiO_2_ layers were used as a bottom gate and gate dielectric, respectively. To make a better back-gate contact, after removing the native oxide on the silicon substrate by dipping in buffer oxide etch (BOE) solution (6:1 volume ratio of 40% NH_4_F in water to 49% HF in water), a 100 nm-thick Au film was sputtered onto the Si substrate. Then, source and drain electrodes were deposited using photolithography followed by electron-beam evaporation of Ti/Au (5 nm/95 nm). The channel length (L) of the transistor varies from 2–14 μm and the channel width (W) is 2 mm, providing maximum channel area of 28 × 10^3^ *μm*^2^. Next, interferometric lithography was performed on the fabricated FET. A negative tone-resist (NR7-500PY) with nominal thickness 500 nm was spun on the sample, followed by two IL exposures using a 355-nm tripled YAG laser source at an incidence angle θ = 30° with a 90° rotation of the sample. The laser exposure time was 10 seconds, with pulse rate of 60 Hz and pulse energy of 100 mJ. After a hard bake at 110° for 60 seconds, the sample was developed in an MF-321 developer for 30 seconds and subsequently a 2D hole array pattern was made in the PR. Optimized O_2_ plasma etching (O_2_ flow, 10 sccm; power, 100 W; pressure, 200 mTorr) was performed for 80 seconds to reduce the PR linewidth and remove graphene in selected areas. The PR/GNM lateral etch rate was 0.8 nm/sec and the vertical etch is estimated to be 1.8 nm/sec. This etching recipe resulted in significant reduction in the PR width, while the PR thickness was only reduced by ~30 percent. Once the etching process is complete, the PR is removed by sample soak in acetone to obtain the final GNM. The samples were annealed at 300 °C in forming gas environment (5% H_2_, 95% N_2_) for 30 min to remove/reduce the polymer resist from the etching mask, and other types of impurities on the mesh surface.

### Device characterization

The electronic properties of mesh-patterned graphene devices were characterized by a JANIS ST-500 micro-manipulated probe station under vacuum (10^−5^ Torr) to eliminate/reduce the hole doping effects due to absorption of oxygen and water molecules at the graphene surface. The probe station was equipped with a Scientific Instruments M9700 temperature controller, and the measurements were carried out with a Keithley 2400 source measure unit (SMU) and Keithley 238 high-current SMU. For comparison purposes, the GNM can be approximated as a mesoscopic honeycomb network of GNR in which the ribbons are interconnected between larger graphene islands. Therefore, the electron and hole mobilities of the GNM were estimated using the formula *μ* = (*gL*/*V*_*ds*_*C*_*ox*_*W*), where g is the transconductance (Figure S5), L is the channel length, *V*_*ds*_ is the source-drain potential, *C*_*ox*_ is the gate capacitance per unit area, and W is the width of channel. *C*_*ox*_ = (*ε*_0_*ε*_*r*_/*d*), where *ε*_0_ is the vacuum permittivity, *ε*_*r*_ and d are the dielectric constant and thickness of the SiO_2_ dielectric layer. It should be noted that in order to study the GNM mobility more accurately, the fringe effect at the ribbon edges of the GNMs and also the exact capacitance of the transistor must be considered, which requires a simulation model based on finite element analysis. SEM imaging was performed on a JEOL- 6500 field-emission microscope. The Raman experiment was carried out by focusing a 532 nm excitation light (output of laser diode) through a dry objective with numerical aperture 0.95. Prior to the Raman studies, the samples were annealed in forming gas environment (5% H_2_, 95% N_2_) to remove polymer resist from the etching mask, and other types of impurities existed on the mesh surface. The scattered light is collected using the same objective and is directed to a CCD spectrometer (Princeton instruments, IsoPlane). The AFM (Neaspec GmbH Inc.) was operated in tapping mode with resonance frequency of cantilever ~250 kHz and tapping amplitude ~50 nm. An ultra-sharp AFM tip (Hi’Res-C14/Cr-Au) with a spike radius of 1 nm was used. Statistical analysis on the acquired AFM images was carried out in AutoCAD software with careful tip corrections.

## Additional Information

**How to cite this article**: Kazemi, A. *et al.* Large-Area Semiconducting Graphene Nanomesh Tailored by Interferometric Lithography. *Sci. Rep.* **5**, 11463; doi: 10.1038/srep11463 (2015).

## Supplementary Material

Supplementary Information

## Figures and Tables

**Figure 1:** The overall fabrication route of GNM, based on interferometric lithography and O_2_ plasma etching. (**a**) SL-CVD graphene on 285 nm-thick SiO_2_ layer and P + Si substrate. (**b**) The sample is covered with a spin-coated negative photoresist (PR). A square 2D hole array pattern is made in the PR by IL. (**c**) To define the mesh structure, an isotropic O_2_ plasma etching is performed at high pressures. During the O_2_ plasma step, the PR line width is reduced, which leads to a decrease in the graphene width under the photoresist. (**d**) The PR mask is removed after a brief soak in acetone solution.

**Figure 2:** SEM images demonstrate the effect of etching on the PR/GNM line-width. (The scale bar for (a) is 100 nm; all the other scale bars are 1 μm). (**a**) Side view image of the PR hole array mask patterned on graphene film after the IL exposure, soft bake, and develop. The nominal PR width above the graphene film is ~70 nm. (**b**) Top view image of the PR hole array mask. (**c**) PR pattern after O_2_ plasma applied for 30 seconds. Due to the high pressure, the etching process was found to be dominantly lateral. The PR width is ~50 nm. (**d**) PR pattern after O_2_ plasma applied for 60 seconds, PR width ~30 nm. (**e**) Final step of etching when the PR width is reduced to ~10 nm after 80 seconds of etching. (**f**) Large-scale top-view image of the PR pattern after 80 seconds of etching. This pattern is continuously written across a 1 × 1 cm^2^ wafer. (**g**) PR/GNM width as a function of the etching duration (blue solid diamonds). The red line is a fit of the experimental data.

**Figure 3:** AFM images of the narrowest GNM and statistical analysis of the neck widths. (**a**–**c**) AFM images acquired from three different spots on the GNM sheet etched for 80 seconds. Insets in **a**–**c**, show high-magnification images. (**d**–**f**) Histograms of neck widths for **a**–**c** fitted with a Gaussian function.

**Figure 4:** Raman Spectra of single-layer CVD GNM. (**a**) Raman spectra of the GNM films with different neck widths compared to pristine single-layer graphene. The spectra were offset for clarity. (**b**) Close-up view to the spectrum acquired from a showing the G and D bands for the mesh structures compared to the pristine graphene sheet. (**c**) Inset: G-band peaks acquired from four Raman scans on four different locations on the narrowest GNM sample. The intensity bands are fitted using Gaussian functions. The FWHM and blue shift of the G bands of the Raman spectra acquired from four different locations on the narrowest GNM sample. The G band FWHM is referred to as the left axis while the G band blue shift is referred to as the right axis. Inset shows the G band intensity of the spectra for those four locations.

**Figure 5:** Transfer characteristics of graphene nanomesh. (**a**) A schematic representation of the GNM-FET. The graphene mesh structure with an average neck width of ~10 nm was fabricated on heavily doped silicon substrate coated by 285 nm-thick SiO_2_ layer as the gate dielectric. The channel length L and width W of the GNM-device are 14 μm and 2 mm, respectively. (**b**) *I*_*d*_ versus gate voltage (*V*_*g*_) recorded at different source-drain voltages obtained at room temperature. (**c**) Source-drain current (*I*_*d*_) versus source-drain voltage (*V*_*ds*_) recorded at different gate voltages at room temperature. (**d**) Comparison of *I*_*d*_−*V*_*g*_ for bulk (black dashed line) and GNM-devices (red solid line) at *V*_*ds*_ = −1 mV at room temperature. The current for bulk graphene-device and GNM-device are specified on the left and right axis, respectively.

**Figure 6:** Temperature study of GNM transfer characteristics. Comparison of *I*_*d*_−*V*_*g*_ curves of the GNM-FET with ~10 nm neck width recorded at *V*_*ds*_ = −1 V and at different temperatures 300, 200, 120, and 77 K.

**Table 1:** Comparison of dimensions and electronic properties of GNMs fabricated by different techniques.

Properties	Fabrication Technique						
	Block Copolymer Litho^20^	Block Copolymer Litho^21^	Nano Imprint Litho^36^	Aluminum Oxide Templating^37^	Nano-Sphere Litho^57^	Nano-Sphere Litho^58^	Interferometric Litho^1^
Graphene type	SL*/MLϒ	SL	SL	SL	N.RŦ	SL	SL
Sheet coverage (*μm*^2^)	N.R	10^6^	4	N.R	N.R	N.R	10^8^
Min neck width (nm)	5	18	7	15	20	65	10
ON/OFF Ratio?	100	39	80	10	10	2	35
Mobility? (*cm*^2^/V.S)	N.R	>1	1000	N.R	N.R	31	80
Band gap? (meV)	100	102	N.R	N.R	N.R	0	30
Channel width (μm)	3	N.R	2	5.8	1.5	1	2
Channel length (μm)	2.3	N.R	2	2	20	2	2000

^1^Present work.

^*^Single layer graphene.

^ϒ^Multilayer/Few Layer graphene.

^Ŧ^Not reported.

^?^At room temperature. Note that the ON/OFF current ratio is a function of source-drain voltage (*V*_*ds*_), and to obtain a reasonable comparison, one should look at the ratios at the same *V*_*ds*_.
